# The Diagnostic Dilemma of Sarcoidosis: A Case of Acute Hypercalcemia

**DOI:** 10.7759/cureus.10399

**Published:** 2020-09-11

**Authors:** Vani Mulkareddy, Varun Bhalla, Soham Upadhye, Preeti Siddam

**Affiliations:** 1 Internal Medicine, Rochester Regional Health, Rochester General Hospital, Rochester, USA

**Keywords:** sarcoidosis, acute hypercalcemia, noncaseating granuloma

## Abstract

Hypercalcemia is a common clinical laboratory abnormality with a majority of cases attributed to malignancy or hyperparathyroidism. Although hypercalcemia is a common manifestation of sarcoidosis, it is rarely the initial presentation. Here we present a case of acute hypercalcemia in a 60-year-old gentleman, which was diagnosed as sarcoidosis following an elaborate workup, including radiological assessment and multiple organ biopsies. This case highlights the diagnostic dilemma of sarcoidosis due to varying clinical presentation that can mimic multiple conditions, including malignancy. Biopsy showing noncaseating granulomas is pathognomic of sarcoidosis. Due to its multisystemic and nonspecific presentation, selecting an appropriate biopsy site is key to diagnosis.

## Introduction

Sarcoidosis is an inflammatory multisystem disease, histologically characterized by noncaseating granulomas. Over 90% of cases have lung involvement; however, 30% of patients can have extrapulmonary manifestations [1]. Presentation varies from asymptomatic cases to organ failure. Sarcoidosis makes up 1% of cases of hypercalcemia [2]. Although a common manifestation of sarcoidosis, hypercalcemia is rarely the initial presentation. Sarcoidosis, like other granulomatous diseases, can clinically and radiologically mimic multiple conditions including multiple myeloma and lymphoma. Due to its vague presentation, diagnosis is often difficult and delayed. Here we present a case of sarcoidosis presenting with acute hypercalcemia in a 60-year-old male. The initial presentation raised concerns for malignancy. Despite radiological evaluation and numerous organ biopsies, the diagnosis remained elusive. Eventual inguinal lymph node biopsy showed noncaseating granulomas diagnostic of sarcoidosis. Treatment of corticosteroids resulted in clinical improvement.

## Case presentation

A 60-year-old Caucasian gentleman with a past medical history significant for hypertension and diabetes presented to his primary care physician with abdominal pain for one month. The pain was insidious in onset and associated with poor oral intake, nausea, and vomiting. His diet had been restricted to clear liquids due to unremitting nausea and vomiting, resulting in 32 pounds of weight loss. He denied recent sick contacts, diarrhea, fever, chills, dysuria, or hematuria. Family and social history were insignificant. Examination revealed a blood pressure of 177/94 mmHg, a pulse rate of 87 beats per minute, afebrile, and epigastric tenderness with no other focal systemic findings.

Initial laboratory workup revealed hemoglobin of 10 mg/dL, platelet count of 250,000 cell/µL, creatinine of 3.32 mg/dL (baseline creatinine 1.13 mg/dL), calcium of 13.8 mg/dL, and phosphorous of 2.5 mg/dL. Initial evaluation for hypercalcemia revealed low parathyroid hormone (PTH) level of 11.3 pg/mL, parathyroid hormone-related peptide (PTHrP) of 1 pmol/L, 25-hydroxyvitamin D level of 17 ng/mL, and a 1,25-dihydroxyvitamin D level elevated to 68 pg/mL. The constellation of abdominal pain, anemia, acute kidney injury, and hypercalcemia guided further evaluation for multiple myeloma. Serum protein electrophoresis and urine protein electrophoresis revealed no monoclonality. Serum immunofixation revealed imperceptible free lambda light chains and elevation in both kappa and lambda free light chains with a ratio of 1.73. A bone marrow biopsy revealed normal cellularity, no significant increase in plasma cells, and no plasma monoclonality. He was started on intravenous fluids, pamidronate, and calcitonin for hypercalcemia. Due to worsening renal function, a renal biopsy was obtained which revealed acute tubular injury with chronic and subacute thrombotic microangiopathy, but no evidence of multiple myeloma or sarcoidosis. He was briefly started on steroids for possible sarcoidosis with improvement in serum calcium; however, a normal serum angiotensin-converting enzyme (ACE) level and lack of granulomas on biopsy arrested concerns for sarcoidosis. Due to microangiopathy on renal biopsy, workup including autoimmune antibody, rheumatoid factor, anti-double-stranded DNA antibody, anti-Sjogren's syndrome A (anti-SSA) antibody, anti-Sjogren's syndrome B (anti-SSB) antibody, and lactate dehydrogenase were all negative. CT of his chest revealed small bilateral pleural effusions and pulmonary edema (Figure 1). CT abdomen revealed enlarged inguinal lymph nodes that were thought to be reactive.

**Figure 1:** CT chest showing bilateral pleural effusions (black arrows) and pulmonary edema.

His calcium and creatinine improved with a dose of denosumab, and he was discharged home with outpatient follow-up. However, due to rising outpatient calcium levels a positron emission tomography (PET) scan was obtained, which revealed multiple tiny fluorodeoxyglucose (FDG)-avid lymph nodes in the chest, abdomen, and pelvis, as well as abnormal FDG labeling in the liver and spleen. Due to concerns for lymphoma, he underwent biopsy of an inguinal lymph node which revealed noncaseating granulomas with giant cells (Figure 2). He was diagnosed with extrapulmonary sarcoidosis, and was subsequently started on steroids with improvement in his hypercalcemia.

**Figure 2:** Inguinal lymph node biopsy showing multiple noncaseating granulomas (black arrows)

## Discussion

Calcium ions play an important role in cellular function, physiological processes, cardiac contractility, and blood coagulation. Therefore, the extracellular concentration of calcium is tightly regulated through feedback mechanisms that involve PTH and 1,25-dihydroxyvitamin D. Integrating signals from the kidney, parathyroid gland, bone, and intestine orchestrate the regulating mechanisms of calcium.

In healthy individuals, vitamin D is stored as a provitamin D in the skin within the epidermis and dermis. Ultraviolet light from the sun converts it into a biologically inactive previtamin D. This previtamin D is enzymatically activated by a two-step hydroxylation reaction in the liver and kidney respectively to 1,25-dihydroxyvitamin D. Vitamin D and its potent metabolites increase extracellular calcium concentration by increasing intestinal epithelial calcium absorption and increased bone resorption through osteoclast production. Though PTH and hypophosphatemia stimulate and enhance renal 1-hydroxylase enzyme; 1, 25 dihydroxyvitamin D in turn inhibits the secretion of PTH, providing a negative feedback regulation.

The cause and pathogenesis of hypercalcemia can be understood based on derangements in normal physiological regulation. Broadly based on the inciting mechanism, hypercalcemia is classified into PTH-dependent and independent causes. The most common causes of hypercalcemia include PTH-dependent hyperparathyroidism and malignancy which causes a PTH-independent hypercalcemia through PTHrP. Although rare, chronic granulomatous diseases can cause a PTH-independent hypercalcemia through enhanced conversion of 25-hydroxyvitamin D to 1,25-dihydroxyvitamin D. Sarcoidosis alone has been found to be the cause of hypercalcemia in only 1% of patients [2].

Sarcoidosis is a multisystem inflammatory disease histologically characterized by noncaseating granulomas. The disease is seen worldwide with an estimate prevalence of 20 to 60 per 100,000 population [3]. Demographically the incidence of sarcoidosis can aggregate in families and certain races. In the United States, the disease is three to four times more common in African Americans, with a slight female gender predominance [4]. Although sarcoidosis can affect any organ, the lung is involved in more than 90% of cases; however, approximately 30% of patients have extrapulmonary manifestations [1,4]. Lymphadenopathy is a hallmark feature, commonly affecting hilar or mediastinal lymph nodes.

Despite advances in immunopathogenesis, the exact etiology of sarcoidosis remains elusive. The formation of the characteristic sarcoid granuloma involves a complex interplay between immune cells and their mediators. These granulomas can produce 1,25-dihydroxyvitamin D independent of PTH. This has been shown through studies of increased calcitriol in an anephric patient with sarcoidosis, in vitro studies of alveolar macrophages and lymph node tissues which showed increased 1,25-dihydroxyvitamin D, as well as increased 1-hydroxylase RNA in alveolar macrophages from patients with sarcoidosis [5-7]. In sarcoidosis, granulomas lack the negative feedback mechanism resulting in unregulated hypercalcemia and hypercalciuria. Elevated PTHrP levels in cases reports of sarcoidosis and other granulomatous diseases along with increased PTHrP expression in bone marrow samples may indicate a role of PTHrP in the pathogenesis of hypercalcemia as well [8].

Diagnosis of sarcoidosis can be challenging when hypercalcemia is the presenting symptom. Although hypercalcemia is a well-studied electrolyte abnormality in sarcoidosis, it is seen in 10% of cases, with severe hypercalcemia of more than 14 mg/dL rarely reported [3]. The incidence of hypercalcemia as the presenting symptom is 3%, with a higher incidence in Caucasian males [1]. As hypercalcemia is a common electrolyte abnormality, all cases must be thoroughly evaluated with PTH, 25-hydroxyvitamin D, and PTHrP to rule out common etiologies. 1,25-dihydroxyvitamin D testing is key to diagnosis as patients with sarcoidosis can have varying levels of 25-hydroxyvitamin D. A subset of patients may be deficient in 25-hydroxyvitamin D [9]. Diagnosis of sarcoidosis in hypercalcemic patients is difficult as the presentation may mimic other granulomatous diseases and malignancies. The presentation of acute kidney injury, anemia, and hypercalcemia in the patient reported above initially raises clinical suspicion of multiple myeloma. Lymphoma was also high on the differential when further evaluation showed diffuse lymphadenopathy on PET scan. Although sarcoidosis was considered in the differential, inconclusive bone marrow biopsy, kidney biopsy, and normal ACE level delayed initial diagnosis. The eventual lymph node biopsy showing noncaseating granulomas was key in clenching the diagnosis, highlighting the importance of selecting the appropriate site to sample. Since sarcoid like histopathological changes can be seen in lymph nodes of patients with neoplastic diseases, caution must be advised while evaluating granulomas in patients without typical features of sarcoidosis. Multiple serological markers, including ACE, serum amyloid A, soluble interleukin-2 receptor, and adenosine deaminase, have been studied, but no clear evidence suggests their utility in diagnosis or disease monitoring. Though elevated ACE levels are seen in 75% of patients with sarcoidosis, ACE can be elevated in other causes of hypercalcemia, including PTH-dependent and oncological-related causes [10,11].

Treatment of hypercalcemia in sarcoidosis consists mainly of corticosteroids. Furthermore, hypercalcemia is an indication to start steroid therapy even in the presence of only mild symptoms. However, other causes of granulomatous diseases including histoplasmosis and tuberculosis should be ruled out prior to steroids. Although steroids are the mainstay of treatment in sarcoidosis, they play an important role in managing hypercalcemia by inhibiting macrophage 1-hydroxylase activity [12]. They reduce the absorption of calcium from the gastrointestinal tract and inhibit osteoclast activity [12]. Additional supportive treatment includes intravenous hydration and loop diuretics to promote renal excretion of calcium. In chronic hypercalcemia of sarcoidosis, patients are advised to avoid sun exposure and reduce fish oil supplementation as they are rich sources of vitamin D. In cases of steroid-resistant sarcoidosis, ketoconazole may be effective in treating hypercalcemia as it inhibits cytochrome P450 enzymes, including 1-hydroxylase [13]. Ketoconazole has also been reported to decrease the use of high-dose corticosteroids. Some case series report promising results with anti-tumor necrosis factor monoclonal antibody, infliximab, in treating refractory hypercalcemia [14].

## Conclusions

This case shows an unusual presentation of sarcoidosis, as acute hypercalcemia is rarely the initial manifestation. This highlights the importance of including sarcoidosis in the differential diagnosis, as it has a wide and varying presentation. As biopsy is key to diagnosis, locating an appropriate site to biopsy is crucial as sarcoidosis can have a multisystemic involvement. In the setting of high clinical suspicion along with elevated 1,25-dihydroxyvitamin D and corticosteroid response, treatment can be initiated while awaiting histological confirmation.
